# Role of T1 Ratio of Marrow, Diffusion-Weighted Imaging, and Chemical Shift Imaging in Multiparametric MRI of the Spine in Spinal Tuberculosis

This article has been retracted.

**DOI:** 10.7759/cureus.91873

**Published:** 2025-09-08

**Authors:** Muhammad Fahad Idrees, Maryum Tayyab, Muhammad Haider, Maham Mujeeb, Usama Mazhar, Ahmad Nazir Tarar

**Affiliations:** 1 Department of Gariatrics, Walsall Manor Hospital, Walsall, GBR; 2 Department of Acute Medicine, Eastbourne District General Hospital, Eastbourne, GBR; 3 Department of Cardiology, Eastbourne District General Hospital, Eastbourne, GBR; 4 Acute Medical Unit, Walsall Manor Hospital, Walsall, GBR; 5 Department of Geriatrics, Stepping Hill Hospital, NHS Stockport Trust, Stockport, GBR; 6 Department of Internal Medicine, Manchester Royal Infirmary Hospital, Manchester University NHS Foundation Trust, Manchester, GBR

**Keywords:** chemical shift imaging, diffusion-weighted imaging (dwi), multi-parametric mri, spinal tuberculosis, t1 ratio of marrow

## Abstract

Objective

This study aimed to evaluate the role of multi-parametric magnetic resonance imaging (MRI) modalities in enhancing the diagnostic accuracy of spinal tuberculosis and improving the overall clinical approach to this complex condition.

Methodology

A total of 50 patients diagnosed with spinal tuberculosis were enrolled in the study. Multi-parametric MRI sequences, including T1-weighted imaging, diffusion-weighted imaging (DWI), and chemical shift imaging (CSI), were performed to assess marrow involvement, diffusion restriction, and fat content within the lesions. Clinical staging of spinal tuberculosis was conducted based on conventional imaging and clinical parameters. Correlations between MRI findings and disease stage were subsequently analyzed.

Results

The study found that significant alterations in the T1 marrow ratio and low apparent diffusion coefficient (ADC) values on DWI were associated with advanced stages of spinal tuberculosis. CSI revealed the presence of fat within granulomatous lesions more frequently in later stages. Among all modalities, DWI demonstrated the highest diagnostic sensitivity and specificity (90% and 85%, respectively), followed by the T1 marrow ratio and CSI. A statistically significant correlation was observed between MRI parameters and clinical staging, highlighting the value of multi-parametric MRI in disease staging.

Conclusion

Multi-parametric MRI - integrating the T1 marrow ratio, DWI, and CSI - proves to be a valuable, noninvasive tool for the early detection, staging, and monitoring of spinal tuberculosis. The findings indicate that DWI offers the highest diagnostic accuracy, underscoring its importance in evaluating spinal tuberculosis. The study supports the integration of advanced MRI techniques into routine clinical practice for more accurate diagnosis and treatment planning.

## Introduction

Spinal tuberculosis (TB) is a severe and debilitating form of extrapulmonary TB that primarily affects the vertebral bodies and intervertebral discs, leading to progressive structural damage, deformity, and neurological impairment [1]. It remains a significant public health concern in regions with a high prevalence of TB, particularly in Asia and Africa. Accurate and early diagnosis of spinal TB is essential for timely intervention and the prevention of complications such as spinal deformities and neurological deficits.

Traditional diagnostic methods, including clinical examination, radiography, and conventional magnetic resonance imaging (MRI), are valuable; however, they often lack the sensitivity and specificity required to differentiate spinal TB from other spinal pathologies such as malignancies or pyogenic infections [2-5]. These limitations have prompted the exploration of advanced imaging techniques that offer more detailed, reliable, and non-invasive insights into the nature of spinal lesions [6].

Among these advanced modalities, multi-parametric MRI has emerged as a powerful tool in evaluating spinal TB [7]. Multi-parametric MRI integrates multiple imaging sequences to assess the spine from different perspectives, enabling comprehensive tissue characterization and improving the differentiation of TB from other spinal conditions. Key MRI parameters, including the T1 marrow ratio, diffusion-weighted imaging (DWI), and chemical shift imaging (CSI), have shown promise in enhancing the diagnostic accuracy of spinal TB [8-10].

The T1 marrow ratio, derived from T1-weighted sequences, is critical in evaluating bone marrow involvement. It reflects alterations in marrow fat and edema, common findings in tubercular infection [11]. This parameter provides insight into the inflammatory activity and can suggest abscess formation, offering crucial information on the extent and progression of disease [12,13].

DWI, sensitive to the movement of water molecules, is particularly valuable in evaluating tissue cellularity and integrity in TB lesions. In spinal TB, DWI highlights areas of restricted diffusion corresponding to abscesses or granulation tissue with high cellular density [14,15]. The apparent diffusion coefficient (ADC), a quantitative measure derived from DWI, assists in differentiating active lesions from chronic or inactive disease and from other mimicking conditions [16].

CSI is another advanced MRI technique that exploits differences in the magnetic properties of fat and water to improve tissue differentiation. In spinal TB, CSI aids in identifying fat necrosis within granulomatous or abscessed regions, contributing to more accurate lesion characterization [17,18].

Integrating these advanced techniques into a multi-parametric MRI approach allows a more nuanced understanding of spinal TB. The combined use of T1 marrow ratio, DWI, and CSI enhances early detection, facilitates treatment monitoring, and supports more informed clinical decision-making [19].

This study aimed to evaluate the role of multi-parametric MRI modalities, including T1 marrow ratio, DWI, and CSI, in enhancing the diagnostic accuracy and staging of spinal TB. It focused on correlating imaging findings with disease extent and assessing the relative performance of different parameters.

## Materials and methods

Study design

This study included individuals with clinically suspected spinal TB who were referred for MRI evaluation at a tertiary care hospital specializing in infectious diseases and spinal disorders. Participants were selected based on a comprehensive set of inclusion criteria: (1) clinical features suggestive of spinal TB, such as back pain, neurological deficits, and positive TB screening tests; (2) absence of primary or metastatic spinal tumors; and (3) provision of informed consent. Patients with contraindications to MRI, such as metallic implants, pacemakers, or pregnancy, were excluded to ensure safety and imaging quality.

Population and sample collection

A convenience sample of 50 eligible patients, aged 3 to 70 years, was included in the study. The sample size was determined using power analysis to ensure adequate statistical power for detecting significant differences in MRI parameters (T1 marrow ratio, DWI, and CSI) across various stages of spinal TB. Each patient underwent a comprehensive MRI protocol comprising conventional sequences (T1-weighted and T2-weighted) as well as advanced imaging sequences, including DWI and CSI. Multi-parametric MRI scans were acquired at predefined intervals - at initial diagnosis and during follow-up - to facilitate longitudinal assessment of disease progression and treatment response.

Data collection

MRI data were acquired using a 3T scanner. The following acquisition parameters were applied: T1-weighted images (TR 500-600 ms, TE 10-15 ms, slice thickness 4 mm, field of view 280-320 mm); T2-weighted images (TR 3,500-4,000 ms, TE 90-100 ms, slice thickness 4 mm, field of view 280-320 mm); DWI with b-values of 0, 500, and 800 s/mm² with automatic ADC map generation; and CSI dual-echo gradient sequences with TE 2.1 ms (in-phase) and 4.2 ms (out-of-phase), TR 120-150 ms. The T1 marrow ratio was calculated by comparing normal and affected vertebral bone marrow signal intensities, using specialized software for accurate segmentation and ratio computation. DWI was performed using standardized b-values to evaluate water diffusion in spinal lesions, and ADC maps were generated for quantitative analysis. CSI sequences determined the fat-to-water ratio within spinal lesions, enabling differentiation between fat-containing granulomas or abscesses and purely fluid-filled collections. Two radiologists with expertise in musculoskeletal TB independently reviewed all MRI scans, and interobserver agreement was assessed using Cohen’s kappa statistics.

Clinical staging criteria

Patients were staged into two categories - early and advanced - based on a composite system integrating conventional imaging and clinical parameters. The reference standard included radiological severity (extent of vertebral destruction, paravertebral/epidural abscess, and deformity) and clinical status (neurological deficits, pain severity, and systemic features). Early stage disease was defined as minimal vertebral involvement without collapse, with absent or small paravertebral abscesses and intact neurology. Advanced stage disease was defined as moderate-to-severe vertebral destruction, presence of large paravertebral/epidural abscesses, spinal deformity, and/or neurological compromise.

Statistical analysis

Descriptive statistics were used to summarize patient demographics and imaging findings. Normality of data distribution was tested using the Shapiro-Wilk test. Continuous variables were expressed as means ± standard deviations or as medians with interquartile ranges, as appropriate. Categorical variables were presented as frequencies and percentages. Correlations between MRI parameters (T1 marrow ratio, ADC values, and fat-to-water ratio) and the clinical stage of spinal TB were analyzed using Pearson or Spearman correlation coefficients, depending on data distribution. Comparisons between early and advanced stages of disease were performed using independent t-tests or Mann-Whitney U tests. Interobserver agreement was quantified using Cohen’s kappa values. A p-value of <0.05 was considered statistically significant. All analyses were conducted using SPSS Version 25.0 (IBM Corp., Armonk, NY, USA).

## Results

As summarized in Table 1, the study enrolled 50 participants, with a mean age of 36.4 ± 12.3 years. Most participants were male, 32 (64%), reflecting the general demographic trend in spinal TB. Back pain was the most common symptom, reported in 50 (100%) cases, followed by weight loss in 30 (60%) and fever in 24 (48%) patients. Neurological deficits were noted in 18 (36%) cases, indicating the severity of spinal involvement in a subset of patients. The duration of symptoms before diagnosis ranged from 3 to 12 months, with an average of 6.5 ± 3.1 months, underlining the chronic nature of spinal TB.

**Table 1:** Demographic and clinical characteristics of participants TB, tuberculosis

Characteristic	N = 50
Age (years)	36.4 ± 12.3
Gender	
Male	32 (64%)
Female	18 (36%)
Duration of symptoms (months)	6.5 ± 3.1
Presenting symptoms	
Back pain	50 (100%)
Neurological deficits	18 (36%)
Fever	22 (44%)
Weight loss	30 (60%)
Comorbidities	
Diabetes	12 (24%)
Hypertension	8 (16%)
Previous TB history	7 (14%)

Table 2 shows the evaluation of the marrow's T1 ratio. Overall, 15 (30%) patients exhibited a normal ratio of 1:1, indicating little or no alteration in marrow signal. Mild alterations (1:1.5) were observed in 20 (40%) patients, while 15 (30%) had significant alterations with a ratio of 1:2 or greater, suggesting marked marrow involvement. DWI revealed that 12 (24%) patients had normal ADC values, indicative of normal tissue integrity. In contrast, 18 (36%) showed mild diffusion restriction (ADC values between 0.7 and 1.0), and 20 (40%) cases exhibited severe restriction (ADC values <0.7), signifying higher cellularity and abscess formation associated with active TB. CSI revealed no fat content in 22 (44%) lesions, mild fat content in 18 (36%), and significant fat content in 10 (20%). The presence of fat content was more commonly observed in advanced stages, correlating with granuloma formation and necrotic tissue within the lesions.

**Table 2:** MRI findings (multi-parametric MRI analysis) ADC, apparent diffusion coefficient values

MRI parameter	Finding	Total number, N (%)
T1 ratio of marrow	Normal (1:1 ratio)	15 (30%)
	Mild alteration (1:1.5)	20 (40%)
	Severe alteration (1:2 or greater)	15 (30%)
Diffusion-weighted imaging	Normal ADC values	12 (24%)
	Mild restriction (ADC 0.7–1.0)	18 (36%)
	Severe restriction (ADC <0.7)	20 (40%)
Chemical shift imaging	No fat content in lesion	22 (44%)
	Mild fat content	18 (36%)
	Significant fat content	10 (20%)

Table 3 depicts that a significant difference was observed in the T1 ratio of marrow between early stage (1.2 ± 0.2) and advanced stage (1.5 ± 0.3) spinal TB (p = 0.02), suggesting that marrow involvement became more pronounced as the disease progressed. Similarly, ADC values from DWI were significantly lower in the advanced stage (0.6 ± 0.2) compared to the early stage (1.2 ± 0.1) (p < 0.001), reflecting increasing diffusion restriction due to abscess formation and higher cellularity. CSI detected that fat content was significantly more prevalent in advanced stages (p = 0.03), correlating with necrotic tissue and granulomas.

**Table 3:** Correlation between MRI parameters and clinical stage of spinal tuberculosis T1 ratio of marrow, T1-weighted signal intensity ratio of bone marrow; DWI (ADC), diffusion-weighted imaging (apparent diffusion coefficient); fat content (CSI), fat content measured by chemical shift imaging

MRI parameter	Early stage (n=20)	Advanced stage (n=30)	p-Value
T1 ratio of marrow	1.2 ± 0.2	1.5 ± 0.3	0.02
ADC (DWI)	1.2 ± 0.1	0.6 ± 0.2	<0.001
Fat content (CSI)	None	Present	0.03

Table 4 summarizes the diagnostic accuracy of the multi-parametric MRI parameters. The T1 ratio of marrow demonstrated a sensitivity of 85% and a specificity of 70%, making it a useful, though not definitive, parameter for diagnosing spinal TB. DWI with ADC values showed the highest diagnostic performance, with a sensitivity of 90% and specificity of 85%, indicating its strong ability to detect active disease. CSI, although practical, showed a lower sensitivity of 75% but a high specificity of 80%, particularly in identifying fat-containing lesions that are characteristic of more advanced disease.

**Table 4:** Diagnostic performance of multi-parametric MRI parameters T1 ratio of marrow, T1-weighted signal intensity ratio of bone marrow; DWI (ADC), diffusion-weighted imaging (apparent diffusion coefficient); fat content (CSI), fat content measured by chemical shift imaging

MRI parameter	Sensitivity (%)	Specificity (%)	Positive predictive value (%)	Negative predictive value (%)
T1 ratio of marrow	85	70	80	75
DWI (ADC)	90	85	87	92
Fat content (CSI)	75	80	77	78

## Discussion

The results of this study highlighted the promising role of multi-parametric MRI-incorporating the T1 ratio of marrow, DWI, and CSI-in enhancing the diagnostic and staging capabilities for spinal TB. A detailed analysis of the findings suggests that integrating these advanced imaging modalities provides a comprehensive understanding of the disease, facilitating its differentiation from other spinal pathologies.

The T1 ratio of marrow, an indicator of bone marrow involvement, revealed varying degrees of alteration across spinal lesions. A significant proportion of participants exhibited mild-to-severe alterations, which correlated with the clinical stage of spinal TB. Notably, marked alterations were more common in the advanced stages of the disease, underscoring the progressive nature of marrow involvement. These observations are consistent with previous studies, which have associated T1 signal changes with bone destruction, marrow edema, and abscess formation in spinal TB [20]. Bhugaloo et al. similarly reported that alterations in the T1 ratio could help distinguish active TB from other conditions such as metastasis or pyogenic infection, reinforcing the diagnostic relevance of this parameter [21].

Analysis of DWI, based on ADC values, demonstrated a strong correlation with disease stage. This study's severe diffusion restriction - reflected by low ADC values - was predominantly observed in advanced spinal TB, suggesting cellular infiltration, abscesses, and necrotic tissue. This aligns with existing literature indicating that diffusion restriction in spinal TB results from increased cellularity and granulation tissue formation [22]. DWI is a well-established, sensitive imaging modality for detecting active disease and evaluating therapeutic response, as it can reveal early changes in tissue architecture not visible on conventional MRI [23].

CSI significantly differentiated fat-containing lesions from those predominantly of fluid or soft tissue. In this study, fat content was frequently observed in lesions at advanced stages, indicative of granuloma formation - a hallmark of chronic TB. These findings align with those of Morrison et al., who reported that CSI could detect fat within abscesses or necrotic tissues, thereby improving diagnostic precision [24]. The increased presence of fat in later disease stages suggests the potential utility of CSI in staging spinal TB and monitoring treatment progression.

Comparative analysis of MRI parameters and clinical staging revealed significant associations. The T1 marrow ratio demonstrated a progressive increase in alteration with disease advancement, as also noted by Unger et al. [25] and Chan et al. [26], who showed that MRI signal intensities correlate with the extent of spinal involvement. The inverse relationship between ADC values and disease stage supports prior research findings, where lower ADC values were linked to higher cellularity and active inflammation [27].

In this study, the diagnostic accuracy of multi-parametric MRI was notably high, especially in the case of DWI. ADC-based DWI exhibited the highest sensitivity and specificity among the parameters, affirming its critical role in detecting active disease. These findings are consistent with evidence demonstrating DWI’s superior performance in identifying early infections and distinguishing tuberculous from non-tuberculous lesions [28]. Although CSI had relatively lower sensitivity, its high specificity enhances its utility in confirming fat-containing granulomatous lesions, contributing additional diagnostic confidence.

Overall, this study suggests that multi-parametric MRI - combining the T1 marrow ratio, DWI, and CSI - provides a more accurate, comprehensive, and noninvasive approach to evaluating spinal TB compared to conventional MRI alone. Integrating these advanced imaging modalities may enable earlier diagnosis, better disease staging, and more effective monitoring of treatment response, ultimately improving clinical management. These results support earlier studies that emphasized the diagnostic benefits of multi-parametric imaging in spinal infections [9,15,16].

Limitations

This study has several limitations. The relatively small sample size and single-center setting may limit the generalizability of the findings to broader populations. The lack of histopathological confirmation in all cases introduces a risk of misclassification of some lesions. Although detailed MRI protocols were followed, the absence of complete acquisition parameters and explicit reproducibility measures across centers may restrict external replication. The exclusive reliance on MRI without incorporating complementary imaging modalities such as CT or PET further limits the comprehensiveness of disease assessment. Finally, the cross-sectional study design restricts the ability to evaluate longitudinal outcomes or prognostic implications, and thus the results should be interpreted within this context.

Despite these limitations, the study demonstrates essential strengths, including the novel application of multi-parametric MRI (T1 marrow ratio, DWI, and CSI) in spinal TB, correlation with clinical staging, and its potential utility as a non-invasive diagnostic and staging tool in routine clinical practice.

## Conclusions

Multi-parametric MRI, incorporating the T1 marrow ratio, DWI, and CSI, shows promise as a valuable tool in assessing spinal TB. Its ability to visualize and quantify distinct aspects of the disease, such as marrow involvement, cellular density, and fat content, suggests potential for enhancing diagnostic accuracy and staging. While our findings support the clinical relevance of these advanced imaging techniques, larger multicenter studies with histopathological confirmation and longitudinal follow-up are warranted before firm conclusions regarding their impact on patient outcomes can be drawn.
